RETRACTED

# Downregulation of lncRNA ZNF582-AS1 due to DNA hypermethylation promotes clear cell renal cell carcinoma growth and metastasis by regulating the N(6)-methyladenosine modification of MT-RNR1

**DOI:** 10.1186/s13046-021-01889-8

**Published:** 2021-03-10

**Authors:** Wuping Yang, Kenan Zhang, Lei Li, Yawei Xu, Kaifang Ma, Haibiao Xie, Jingcheng Zhou, Lin Cai, Yanqing Gong, Kan Gong

**Affiliations:** 1 Department of Urology, Peking University First Hospital, No. 8, Xishiku Street, Xicheng District, Beijing, 100034 China; 2 Hereditary Kidney Cancer Research Center, Peking University First Hospital, No. 8, Xishiku Street, Xicheng District, Beijing, 100034 China; 3 Institute of Urology, Peking University, Beijing, 100034 P. R. China; 4 National Urological Cancer Center, Beijing, 100034 P. R. China

**Keywords:** ccRCC, ZNF582-AS1, DNA methylation, N(6)-methyladenosine modification, MT-RNR1

## Abstract

**Background:**

Emerging evidence confirms that lncRNAs (long non-coding RNAs) are potential biomarkers that play vital roles in tumors. ZNF582-AS1 is a novel lncRNA that serves as a potential prognostic marker of cancers. However, the specific clinical significance and molecular mechanism of ZNF582-AS1 in ccRCC (clear cell renal cell carcinoma) are unclear.

**Methods:**

Expression level and clinical significance of ZNF582-AS1 were determined by TCGA-KIRC data and qRT-PCR results of 62 ccRCCs. DNA methylation status of ZNF582-AS1 promoter was examined by MSP, MassARRAY methylation and demethylation analysis. Gain-of-function experiments were conducted to investigate the biological roles of ZNF582-AS1 in the phenotype of ccRCC. The subcellular localization of ZNF582-AS1 was detected by RNA FISH. iTRAQ, RNA pull-down and RIP-qRT-PCR were used to identify the downstream targets of ZNF582-AS1. rRNA MeRIP-seq and MeRIP-qRT-PCR were utilized to examine the N(6)-methyladenosine modification status. Western blot and immunohistochemistry assays were used to determine the protein expression level.

**Results:**

ZNF582-AS1 was downregulated in ccRCC, and decreased ZNF582-AS1 expression was significantly correlated with advanced tumor stage, higher pathological stage, distant metastasis and poor prognosis. Decreased ZNF582-AS1 expression was caused by DNA methylation at the CpG islands within its promoter. ZNF582-AS1 overexpression inhibited cell proliferative, migratory and invasive ability, and increased cell apoptotic rate in vitro and in vivo. Mechanistically, we found that ZNF582-AS1 overexpression suppressed the N(6)-methyladenosine modification of MT-RNR1 by reducing rRNA adenine N(6)-methyltransferase A8K0B9 protein level, resulting in the decrease of MT-RNR1 expression, followed by the inhibition of MT-CO2 protein expression. Furthermore, MT-RNR1 overexpression reversed the decreased MT-CO2 expression and phenotype inhibition of ccRCC induced by increased ZNF582-AS1 expression.

RETRACTED

**Conclusions:**

This study demonstrates for the first time that ZNF582-AS1 functions as a tumor suppressor gene in ccRCC and ZNF582-AS1 may serve as a potential biomarker and therapeutic target of ccRCC.

**Supplementary Information:**

The online version contains supplementary material available at 10.1186/s13046-021-01889-8.

## Background

CcRCC (Clear cell renal cell carcinoma) is the most common histological subtype of kidney cancers, affecting more than 403,000 individuals and causing over 175,000 deaths in 185 countries worldwide per year [1]. At present, radical surgical operation is the main treatment for patients with early ccRCC, and targeted therapy may prolong the survival time of patients with advanced or metastatic ccRCC [2–4]. Unfortunately, the prognosis of ccRCC patients is still poor, especially for patients with advanced and metastatic disease, the 5-year survival rate after diagnosis is only 12% [4–6]. Therefore, finding more effective and safer therapeutic targets has great potential value for improving the prognosis of ccRCC patients.

Although ncRNAs (non-coding RNAs) account for more than 90% of human genomic RNA, most of the > 50,000 ncRNAs have only been discovered in the past 10 years and remain largely unstudied [7, 8]. As a new class of ncRNAs, lncRNAs (long non-coding RNAs) are characterized as non-coding transcripts greater than 200 base pairs in length transcribed by RNA Pol II from independent promoters [9]. In many cases, lncRNAs have been proven to be the main regulator of gene expression, thus they can play key roles in a variety of biological functions and disease processes including cancers [10]. Recent accumulating evidence has indicated that lncRNAs, such as OTUD6B-AS1, URRCC, HOTAIRM1 and MRCCAT1, play important regulatory roles in diverse biological processes in ccRCC [11–14].

Epigenetic alterations have been considered as one of the hallmarks of tumorigenesis [15], and emerging evidence suggests that epigenetic modification is one of the main mechanisms regulating lncRNA expression and tissue specificity [16, 17]. For instance, DNA methylation-mediated activation of lncRNA SNHG12 increases temozolomide resistance in glioblastoma [18]; aberrant methylation-mediated downregulation of lncRNA SSTR5-AS1 promotes the progression and metastasis of laryngeal squamous cell carcinoma [19]; LOC134466 methylation accelerates oncogenesis of endometrial carcinoma through LOC134466/hsa-miR-196a-5p/TAC1 axis [20]. Previous studies have reported that ZNF582-AS1 is a novel lncRNA with diagnostic and prognostic values in RCC based on TCGA (The Cancer Genome Atlas) data [21], and it is epigenetically silenced by aberrant DNA methylation in colorectal cancer [22]. However, the specific clinical significance of ZNF582-AS1 in ccRCC and its DNA methylation status and molecular mechanism remain unknown.

RETRACTED

In this study, we found that lncRNA ZNF582-AS1 expression was significantly downregulated in ccRCC tissues than that in the adjacent normal renal tissues, and decreased ZNF582-AS1 expression was significantly correlated with advanced tumor stage, higher pathological stage, distant metastasis, and poor prognosis. Besides, we identified that ZNF582-AS1 was epigenetically deactivated by DNA methylation at the CpG islands within its promoter, which played an important role in decreased ZNF582-AS1 transcription in ccRCC. Moreover, we showed that ZNF582-AS1 overexpression inhibited cell proliferative, migratory and invasive ability, and increased cell apoptosis in vitro and in vivo. Mechanistically, we demonstrated that ZNF582-AS1 overexpression suppressed the N(6)-methyladenosine modification of MT-RNR1 by reducing rRNA adenine N(6)-methyltransferase A8K0B9 protein level, resulting in the decrease of MT-RNR1 expression, followed by the inhibition of MT-CO2 protein expression. Furthermore, we confirmed that MT-RNR1 overexpression reversed the decreased MT-CO2 expression and phenotype inhibition of ccRCC induced by increased ZNF582-AS1 expression. Collectively, our findings demonstrate that ZNF582-AS1 is a powerful tumor biomarker, which highlights its potential clinical value as a promising prognostic and therapeutic target of ccRCC.

## Methods

### Bioinformatic data mining

Level-3 RNA-sequencing data, DNA methylation data, the clinicopathological and survival data of patients with ccRCC were downloaded from The Cancer Genome Atlas-Kidney Renal Clear Cell Carcinoma (TCGA-KIRC) (https://portal.gdc.cancer.gov/). catRAPID, an algorithm, was used to estimate the binding propensity of A8K0B9-ZNF582-AS1 pair (http://service.tartaglialab.com/page/catrapid_group).

### Clinical sample collection

62 fresh ccRCC tissue samples and pair-matched adjacent normal tissue samples were obtained from patients who underwent surgery. After resection, fresh ccRCC and pair-matched adjacent normal renal tissues obtained from the same patient were snap-frozen in liquid nitrogen immediately. This study was approved by the Biomedical Research Ethics Committee of Peking University First Hospital (Beijing, China, IRB00001052–18004), and each patient included in this study signed an informed consent form.

RETRACTED

### Cell culture and transfection

The normal human renal tubular epithelial cell line HK2, human embryonic kidney cell line HEK293 and 5 ccRCC cell lines OSRC2, 786-O, Caki-1, 769-P and A498 were used in this study. HK2, HEK293, Caki-1 and A498 cells were cultured in DMEM supplemented with 10% foetal bovine serum, while the OSRC2, 786-O and 769-P cells were cultured in RPMI 1640 supplemented with 10% FBS.

For overexpression of ZNF582-AS1, A8K0B9, B4DRY2 and MT-RNR1, recombinant pLV-EF1a-hluc-P2A-Puro-WPRE-CMV-ZNF582-AS1, pLV-hef1a-mNeongreen-P2A-Puro-WPRE-CMV-A8K0B9-3Xflag, pLV-hef1a-mNeongreen-P2A-Puro-WPRE-CMV-B4DRY2-3Xflag, pLV-hef1a-Bla-WPRE-CMV-MT-RNR1 and their corresponding control plasmid vectors were constructed by the SyngenTech Company (SyngenTech Co. Ltd., Beijing, China). Cells were transfected with the corresponding vector using Lipofectamine 3000 Transfection Reagent (Invitrogen, USA) according to the manufacturer’s instructions. After 48 h, cells transfected with the corresponding vector were harvested for qRT-PCR. The stable cell line was established by lentivirus infection accordingly. Lenti-virus was produced using three vectors system: transfer vector, viral packaging (psPAX2) and viral envelope (pMD2G) at 6:3:1 ratio transfected into 293 T cells. Then, the cells were infected by lentiviruses according to the MOI value (the number of lentiviruses per number of cells). The ZNF582-AS1, A8K0B9 and B4DRY2 overexpressed stable cell lines were selected with puromycin (5 μg/mL) and MT-RNR1 overexpressed stable cell lines were selected with blasticidin (10 μg/mL).

### Quantitative real-time PCR (qRT-PCR)

Total RNA was extracted from the tissue samples or the transfected cells using the TRIzol reagent (Invitrogen; USA). cDNA was generated using reverse transcription (Invitrogen; USA). qRT-PCR was performed according to the manufacturer’s instructions, and normalized to GAPDH. All experiments were repeated at least three times. The detailed primer sequences included in this study are shown in Additional file 1: Table S1.

### RNA fish

RNA FISH was performed using a fluorescent in situ hybridization kit (RiboBio, China) following the manufacturer’s instructions. The lncRNA ZNF582-AS1, U6 and 18S FISH probes were also designed and synthesized by the RiboBio Company. Fluorescence detection was performed with a confocal laser-scanning microscope (Leica, Germany).

### Methylation-specific PCR (MSP)

MethPrimer 2.0 (http://www.urogene.org/methprimer2/) was used to predict the CpG island of ZNF582-AS1 and designing MSP primers. Genomic DNA was extracted from ccRCC and adjacent normal renal tissues. The purified DNA was exposed to bisulfite with a DNA Bisulfte Conversion Kit (Tiangen, China) according to the manufacturer’s protocol. The methylation-specific PCR (MSP) of bisulfite-transformed DNA was carried out with a nested, two-stage PCR method. Amplified PCR products were separated by 1.5% agarose gel electrophoresis and visualized with GelRed. The specific primers used for MSP were listed in Additional file 1: Table S1.

RETRACTED

### Sequenom MassARRAY quantitative DNA methylation analysis

Genomic DNA was extracted from ccRCC and pair-matched adjacent normal tissues, and the bisulfite conversion reaction was performed according to the manufacturer’s instructions. The PCR mixtures were pre-heated for 4 min at 94 °C, followed by 45 cycles of 94 °C for 20 s, 56 °C for 30 s and 72 °C for 1 min, the final extension at 72 °C for 3 min. PCR products were incubated with Shrimp Alkaline Phosphatase following the manufacturer’s protocol. After in vitro transcription and RNase A digestion, small RNA fragments with CpG sites were acquired for the reverse reaction. The methylation ratios of the products were calculated using Epityper software Version 1.0 (Sequenom, San Diego, CA, USA). The Sequenom MassARRAY platform (Oebiotech, Shanghai, China) was utilized to quantitatively analyze the DNA methylation status of ZNF582-AS1 DNA. PCR primers were designed using EpiDesigner, and their sequences were listed in Additional file 1: Table S1.

### Demethylation analysis

ccRCC cells were seeded in six-well plates at a concentration of 1 × 10^5^ cells per well, grown for 24 h, and then treated with 5 μM 5-Aza-2′-deoxycytidine (5-Aza-dC, A, Sigma-Aldrich) for 4 days. Cells were cultured with or without 100 Nm Trichostatin A (TSA, T, Sigma-Aldrich) for the final 24 h. RNA was isolated for qRT-PCR analysis and DNA was extracted for ZNF582-AS1 MSP.

### Ethynyl-2-deoxyuridine (EdU) incorporation and CCK-8 assays

Cell proliferation was determined by an ethynyl-2-deoxyuridine (EdU) incorporation assay using an EdU Apollo DNA in vitro kit (RiboBio, Guangzhou, China) and BeyoClick™ EdU Cell Proliferation Kit with DAB (Beyotime, China) following the manufacturer’s instructions. ccRCC cells were seeded in 96-well plates and cell viability was evaluated with the Cell Counting Kit 8 (TransGen Biotech, Beijing, China). Absorbance was measured (OD value) at a wavelength of 450 nm.

### TUNEL and flow cytometry assays

Cells apoptosis was detected by TUNEL staining using One Step TUNEL Apoptosis Assay Kit (Beyotime, China) and Colorimetric TUNEL Apoptosis Assay Kit (Beyotime, China) according to the manufacturer’s instructions. Cell apoptosis was also assayed by staining with Annexin V-FITC and PI (KeyGEN BioTECH) following manufacturer’s instructions and detected by a flow cytometer (FACSCalibur, Becton Dickinson, New Jersey, USA).

RETRACTED

### Wound healing assay

Cell migration was determined via a wound-healing assay. Briefly, approximately 3 × 10^5^ cells were seeded in 6-well plates at equal densities and grown to 80% ~ 90% confluency. Artificial gaps were generated by a 1 ml sterile pipette tip after transfection. Wounded areas were marked and photographed with a microscope.

### Transwell migratory and invasive assays

For the transwell migration assay, 2000 cells were plated into the upper chambers (24-well insert, pore size 8 μm, Corning) with 100 μL serum-free PRIM-1640. The lower chambers were filled with 600 μL PRIM-1640 containing 10% FBS. 48 h later, cells under the surface of the lower chamber were washed with PBS and stained with 0.5% crystal violet for 10 min. For the invasion assay, 2000 cells were seeded on transwells coated with 100 μL Matrigel (1:4 dilution in PBS, Corning Inc., USA). The culture conditions were the same as described for the transwell migration assay. After 48 h, adherent cells on the lower surface were stained with 0.5% crystal violet. The number of cells on the lower surface was photographed with a microscope.

### iTRAQ (isotope tagging for relative and absolute protein quantitation)

Protein extraction was carried out using the RIPA buffer (Applygen, China). The BCA protein assay Kit (Applygen, China) was used to quantitate total protein levels. The protein (20 μg) from each sample was mixed with 5X loading buffer and separated on a 12.5% SDS-PAGE gel and visualized by Coomassie Blue R-250 staining. A filter-aided sample preparation (FASP) was used to remove the detergent, DTT, and other low molecular weight components and digest the proteins. One hundred micrograms of each peptide mixture was labeled using an iTRAQ reagent 8-plex kit (SCIEX, Framingham, MA) according to the manufacturer’s instructions. iTRAQ-labeled peptides were fractionated by Phenomenex Luna Strong Cation Exchange (SCX) chromatography. Each fraction was injected for nano-LC-MS/MS analysis. High-resolution LC-MS/MS analysis was performed on a Q Exactive mass spectrometer (Thermo Fisher Scientific) operated in a positive ion mode that was coupled to an EASY-nLC liquid chromatograph (Thermo Fisher Scientific). The MS data were acquired in a data-dependent acquisition mode. The top 20 precursor ions were selected from each MS full scan in the HCD collision cell. The instrument was run with the peptide recognition mode enabled. The raw files were processed using Proteome Discoverer 1.4 (Thermo Scientific) and searched using the Mascot search engine (version 2.2, Matrix Science) against the UniProt protein human database (134,919 sequences). The results were evaluated for difference significance using ANOVA analysis. It is recommended to select proteins with *p* value less than 0.05, ratio ≥ 1.2 or ratio ≤ 0.83 as differential proteins.

RETRACTED

### Western blot analysis

Protein extraction was carried out using the RIPA buffer, and the BCA protein assay Kit was used to quantitate total protein levels. Protein (40 μg per lane) was separated by SDS-PAGE. Proteins were transblotted to PVDF membranes, and membranes were blocked in 5% nonfat milk powder and incubated overnight at 4 °C with anti-FLAG (1:1000; CST, 14793S), anti-TFB1M (1:1000; Sigma-Aldrich, HPA029428), anti-TFB1M (1:1000; Abcam, ab236901), anti-MT-CO2 (1:1000; Abcam, ab79393), Bcl-2 (1:1000, Abcam, ab32124), Cleaved Caspase-3 (1:1000, Affinity, AF7022), E-cadherin (1:1000, CST, 3195 T) and N-cadherin (1:1000, CST, 13116 T). After incubated with horseradishperoxidase-conjugated goat anti-rabbit IgG, membranes were resolved by chemiluminescence. All membranes were stripped and reprobed with anti-GAPDH antibody (1:8000, Proteintech, China) as a loading control.

### Immunohistochemistry staining

The paraffin sections of mice pulmonary metastasis samples were used to perform immunohistochemical staining to measure the protein expression levels of E-cadherin and N-cadherin. The specific primary antibody information is as follows: anti-E-cadherin (1:400, CST, 3195 T) and anti-N-cadherin (1:125, CST, 13116 T).

### RNA pull-down assay

The ZNF582-AS1-binding proteins were examined using RNA pull-down assays according to the instructions of the Pierce Magnetic RNA-Protein Pull-Down Kit (Thermo Fisher Scientific, 20,164, USA). Biotin-labeled RNAs were transcribed in vitro with the Biotin RNA Labeling Mix and T7 RNA polymerase (RiboBio, China). Biotinylated RNAs were mixed with streptavidin magnetic beads (Thermo Fisher Scientific, 20,164, USA) at 4 °C overnight. Total cell lysates were freshly prepared and added to each binding reaction with Protease/Phosphatase Inhibitor Cocktail and RNase inhibitor, and then the mixture was incubated with rotation for 1 h at 4 °C. After washing thoroughly three times, the RNA–protein binding mixture was boiled in SDS buffer and the eluted proteins were detected by western blot.

### RNA immunoprecipitation (RIP) assay

The RIP experiments were performed with a Magna RIP RNA-Binding Protein Immunoprecipitation Kit (17–700, Millipore, USA) according to the manufacturer’s protocol. Cell lysates were prepared and incubated with RIP buffer containing magnetic beads conjugated with human anti-Flag antibody (Sigma Aldrich). Normal mouse IgG (17–700, Millipore) functioned as the negative control. The RNA fraction precipitated by RIP was analyzed by qRT-PCR.

RETRACTED

### rRNA MeRIP-seq and MeRIP-qRT-PCR

Total RNAs were extracted by TRizol from the stable ZNF582-AS1 overexpressed and control OSRC2 cells. RNA was tested for quality using nanodrop and gel electrophoresis. Chemically fragmented RNA (100 nucleotides) was incubated with m6A antibody for immunoprecipitation according to the standard protocol of Magna methylated RNA immune-precipitation (MeRIP) m6A Kit (17–10,499, Millipore, USA). Enrichment of m6A containing rRNA was analyzed either by high-throughput rRNA sequencing or by qRT-PCR with the primers listed in Additional file 1: Table S1.

### Mouse model experiments

Animal experiments were conducted in accordance with the NIH Guidelines for the Care and Use of Laboratory Animals with the approval of the Review Board of Peking University First Hospital, Beijing. Mice were maintained under pathogen-free conditions with regulated temperature and humidity levels. Mice were randomly assigned to cages in groups of 5 and fed ad libitum under controlled light/dark cycles.

Twenty-four 5-week-old male BALB/c nude mice were purchased from Vitalriver, Beijing, China. Approximately 5 × 10^6^ ZNF582-AS1-overexpressed, MT-RNR1-overexpressed-ZNF582-AS1-overexpressed and control OSRC2 cells suspended in 100 μL Hank’s Balanced Salt Solution (Thermo Fisher Scientific, USA) were mixed with Matrigel (1:1, Corning Inc., USA). Then, 200 μL tumor cells were subcutaneously implanted on the right flank of 6-week BALB/c nude mice using a 28-gauge needle (Thermo Fisher Scientific, USA). Tumor size was measured every week and calculated using the formula: (length × width^2^)/2. For cell proliferation assay, ethynyl-2-deoxyuridine (EdU, 50 mg/kg; Beyotime, China) was intraperitoneally injected 4 h before mice were euthanized.

For the metastasis experiment, twenty 5-week-old male B-NDG mice (NOD- *Prkdc*^*scid*^ *IL2rg*^*tm1*^/Bcgen) that lacked mature T cells, B cells, and natural killer (NK) cells, were purchased from BIOCYTOGEN, Beijing, China. Approximately 5 × 10^5^ ZNF582-AS1- -Luc, MT-RNR1-ZNF582-AS1-Luc and or CON-Luc Caki-1 cells were suspended in 150 ul PBS and injected into the lateral tail veins of each unanesthetized B-NDG mouse at five-weeks-old. Thirty days after injection, mice were anesthetized with isoflurane (YIPIN Pharmaceutical CO., LTD, Hebei, China). Ten minutes after D-Luciferin, sodium salt (150 mg/kg) was injected intraperitoneally, and cancer cells were detected with an in vivo imaging system, Xenogen IVIS (PerkinElmer, MA, USA). The total flux in photons per second were calculated and reported for each mouse’s lung and liver region using Living Image 4.3.1 (PerkinElmer/Caliper).

RETRACTED

### Statistical analyses

Non-parametric Mann-Whitney test was used to detect differences in continuous variables. Survival curves for patients were plotted using the Kaplan-Meier method, with log-rank tests for statistical significance. The correlation between ZNF582-AS1 expression and MT-RNR1 expression, MT-RNR1 expression and MT-CO2 mRNA expression in ccRCC was examined using Pearson’s correlation analysis. All data were analyzed using Graphpad prism 7.0 and R language. A *p* value of < 0.05 was regarded as statistical difference.

## Results

### ZNF582-AS1 expression was downregulated in ccRCC

Based on TCGA-KIRC RNA-seq and clinical data, ZNF582-AS1 expression was downregulated in ccRCC tissues compared with in the adjacent normal renal tissues (Fig. 1a), and lower ZNF582-AS1 expression was associated with advanced tumor stage, higher pathological stage, distant metastasis, and shorter OS (Overall Survival) and DFS (Disease Free Survival) (Fig. 1b). To verify these results, we examined the expression of ZNF582-AS1 in 62 paired ccRCC tissues (ccRCC and adjacent normal renal tissues), and the detail clinical information of these 62 ccRCC patients was shown in Table 1. The qRT-PCR results showed that ZNF582-AS1 expression was significantly decreased in 83.9% (52/62) of ccRCC tissues than that in the adjacent normal renal tissues (Fig. 1c, d). Moreover, ZNF582-AS1 expression was significantly lower in advanced tumor stage and distant metastatic ccRCC (Fig. 1e). In addition, we examined ZNF582-AS1 expression in ccRCC cell lines, and results indicated that ZNF582-AS1 expression was generally downregulated in ccRCC cell lines, especially in OSRC2 and Caki-1 cell lines (Fig. 1f). The subcellular localization of lncRNAs is closely related to their biological function and potential molecular roles [23]. Thus, we used RNA FISH to detect the subcellular localization of ZNF582-AS1 in OSRC2 and Caki-1 cell lines, and the RNA FISH results showed that ZNF582-AS1 was distributed mostly in the cytoplasm of ccRCC cells (Fig. 1g).

**Fig. 1:** Expression and clinical significance of ZNF582-AS1 in ccRCC and its subcellular localization in ccRCC cells. **a** ZNF582-AS1 expression was downregulated in ccRCC tissues (*n* = 539) compared with in the adjacent normal renal tissues (*n* = 72) based on TCGA-KIRC data. **b** Lower ZNF582-AS1 expression was associated with advanced tumor stage (T1-T2 (*n* = 340), T3-T4 (*n* = 190)), higher pathological stage (Stage I-II (*n* = 322), Stage III-IV (*n* = 205)), distant metastasis (No (*n* = 440), Yes (*n* = 80)), and shorter OS (*n* = 530) and DFS (*n* = 485) based on TCGA-KIRC data. According to the median cutoff of ZNF582-AS1 expression, patients were divided into two groups for survival analysis. **c** The heights of the columns in the chart represented the log2-transformed fold changes (ccRCC tissue/ adjacent normal renal tissues) in ZNF582-AS1 expression in 62 patients with ccRCC. **d** ZNF582-AS1 expression was decreased in ccRCC tissues compared with in the adjacent normal renal tissues based on qRT-PCR results. **e** ZNF582-AS1 expression was downregulated in advanced tumor stage (T1-T2 (*n* = 41), T3-T4 (*n* = 21)) and distant metastatic (No (*n* = 43), Yes (*n* = 19)) ccRCC patients. **f** ZNF582-AS1 expression was generally decreased in ccRCC cells. **g** Subcellular localization of ZNF582-AS1 in ccRCC cells

**Table 1:** The clinicopathologic characteristics of 62 ccRCC patients

Clinicopathologic characteristics	n(%)
Age	
< 60	33 (53.2)
> =60	29 (46.8)
Tumor size	
< 2 cm	7 (11.3)
> = 2 cm, < 5 cm	40 (64.5)
> = 5 cm	15 (24.2)
Gender	
Male	46 (74.2)
Female	16 (25.8)
Tumor stage	
T1/T2	41 (66.1)
T3/T4	21 (33.9)
Metastasis	
No	43 (69.4)
Yes	19 (30.6)

RETRACTED

### ZNF582-AS1 expression was regulated by DNA methylation in ccRCC

Epigenetic alterations such as promoter CpG methylation can mediate activation of oncogenes and inactivation of tumor suppressor genes to promote tumorigenesis [24]. In the TCGA-KIRC methylation data, the methylation levels of 13 CpG sites of ZNF582-AS1 DNA (cg25267765, cg24733179, cg24039631, cg22647407, cg20984085, cg13916740, cg11740878, cg09568464, cg08464824, cg07778983, cg07135042, cg02763101, cg01772700) were significantly higher in ccRCC compared with adjacent normal renal tissues (Additional file 2: Figure S1 a, b), and the methylation levels of these 13 CpG sites were negatively correlated with ZNF582-AS1 expression (Additional file 2: Figure S1 c). All of these 13 CpG sites were located in the promoter region of ZNF582-AS1 DNA, and the detail information of these CpG sites was shown in Table 2. Besides, the promoter of ZNF582-AS1 is a bidirectional promoter and also codes for a protein-coding gene, ZNF582, which is transcribed in the opposite direction. Thus, ZNF582 expression may mirror the expression of ZNF582-AS1. We tested the correlation between ZNF582 expression and the methylation levels of these 13 CpG sites, and our results indicated that ZNF582 expression was also negatively correlated with the methylation levels of the other 12 CpG sites except cg01772700 (Additional file 3: Figure S2). Moreover, high methylation levels of 10 CpG sites (cg25267765, cg24733179, cg24039631, cg22647407, cg20984085, cg13916740, cg09568464, cg08464824, cg07135042, cg02763101) were associated with poor OS, and high methylation levels of 6 CpG sites (cg22647407, cg13916740, cg09568464, cg08464824, cg07778983, cg02763101) were correlated with poor DFS (Additional file 4: Figure S3 a, b). Thus, the above results determined that DNA hypermethylation might play an important role in the decreased expression of ZNF582-AS1 in ccRCC.

RETRACTED

**Table 2:** The detailed information of 13 CpG sites in ZNF582-AS1 promoter based on TCGA-KIRC data

Composite Element REF	Chromosome	Start	End	CGI_Coordinate	Feature_Type
cg01772700	chr19	56,393,073	56,393,074	CGI:chr19:56393267–56,393,986	N_Shore
cg24733179	chr19	56,393,211	56,393,212	CGI:chr19:56393267–56,393,986	N_Shore
cg11740878	chr19	56,393,386	56,393,387	CGI:chr19:56393267–56,393,986	Island
cg09568464	chr19	56,393,532	56,393,533	CGI:chr19:56393267–56,393,986	Island
cg02763101	chr19	56,393,576	56,393,577	CGI:chr19:56393267–56,393,986	Island
cg22647407	chr19	56,393,596	56,393,597	CGI:chr19:56393267–56,393,986	Island
cg08464824	chr19	56,393,608	56,393,609	CGI:chr19:56393267–56,393,986	Island
cg13916740	chr19	56,393,628	56,393,629	CGI:chr19:56393267–56,393,986	Island
cg24039631	chr19	56,393,644	56,393,645	CGI:chr19:56393267–56,393,986	Island
cg20984085	chr19	56,393,663	56,393,664	CGI:chr19:56393267–56,393,986	Island
cg25267765	chr19	56,393,725	56,393,726	CGI:chr19:56393267–56,393,986	Island
cg07135042	chr19	56,393,783	56,393,784	CGI:chr19:56393267–56,393,986	Island
cg07778983	chr19	56,394,014	56,394,015	CGI:chr19:56393267–56,393,986	S_Shore

To verify the analysis results of TCGA-KIRC methylation data, MethPrimer 2.0 was used to detect the CpG islands in the promoter region of ZNF582-AS1 DNA and design MSP primers (Fig. 2a). MSP results showed that compared with HK2 cells, ZNF582-AS1 DNA was significantly hypermethylated in ccRCC cells, especially in OSRC2 and Caki-1 cell lines (Fig. 2b). Moreover, the MSP results showed that ZNF582-AS1 was significantly hypermethylated in ccRCC tissues than that in the adjacent normal renal tissues (Fig. 2c). Sequenom MassARRAY quantitative DNA methylation analysis was utilized to examine the DNA methylation status of 38 CpG sites in 10 paired ccRCC tissues, including 8 CpG sites detected in TCGA-KIRC methylation data (cg09568464, cg02763101, cg22647407, cg08464824, cg13916740, cg24039631, cg20984085, cg25267765, red mark) (Fig. 2d), and the results showed that the average methylation levels of these 38 CpG sites was significantly higher in ccRCC than that in the adjacent normal renal tissues (Fig. 2e, f, g). Furthermore, ZNF582-AS1 expression was significantly upregulated after 5-Aza-2′-deoxycytidine (5-aza-dC, 5-Aza, A) and Trichostatin A (TSA, T) induced the demethylation of ZNF582-AS1 promoter in OSRC2 and Caki-1 cells (Fig. 2h).

RETRACTED

**Fig. 2:** ZNF582-AS1 expression was regulated by DNA methylation in ccRCC. **a** Detection of CpG islands in ZNF582-AS1 promoter and design of MSP primers. The horizontal axis of the curved lines represents the input sequence of ZNF582-AS1, and the vertical axis of the curved lines represents GC percentage. TSS: Transcription Start Sites. **b** MSP analysis of ZNF582-AS1 promoter DNA methylation status in ccRCC cell lines. **c** MSP analysis of ZNF582-AS1 promoter DNA methylation status in ccRCC tissues. **d** Detection of 38 CpG sites in ZNF582-AS1 promoter. **e** Quantitative detection of DNA methylation level of 38 CpG sites in ZNF582-AS1 promoter using Sequenom MassARRAY quantitative DNA methylation analysis. **f** and **g** Comparison of the DNA methylation levels of 38 CpG sites in ccRCC and adjacent normal renal tissues. **h** Treatment with 5-aza-dC and TSA demethylated ZNF582-AS1 promoter and increased ZNF582-AS1 expression in OSRC2 and Caki-1 cells. T refers to Tumor tissue of ccRCC, N refers to Adjacent normal kidney tissue. M = Methylated, U = Unmethylated

### ZNF582-AS1 overexpression attenuated cell proliferation and induced cell apoptosis in vitro and in vivo

Downregulated ZNF582-AS1 expression and higher ZNF582-AS1 DNA methylation levels were observed in OSRC2 and Caki-1 cells. Then, we generated a lentiviral vector expressing ZNF582-AS1 for a functional study. The effect of ZNF582-AS1 on the growth of OSRC2 and Caki-1 cells was determined using CCK-8 and EdU incorporation assays. Flow cytometry and TUNEL assays were performed to evaluate the apoptosis in the cells. Our results suggested that ZNF582-AS1 overexpression inhibited cell proliferation (Fig. 3a, b, c) and promoted cell apoptosis (Fig. 3d, e, f, g) in OSRC2 and Caki-1 cells. Consistent with the weak proliferative ability and high apoptotic rate observed in the ZNF582-AS1-overexpressed OSRC2 and Caki-1 cells, the xenograft experiment in mice found that ZNF582-AS1-overexpressed tumors grew slower than those in the control group (Fig. 3h, i, j). Moreover, the results of immunohistochemistry confirmed that ZNF582-AS1 overexpression inhibited cell proliferation and promoted cell apoptosis in tumors (Fig. 3k, l).

**Fig. 3:** ZNF582-AS1 overexpression attenuated cell proliferation and induced cell apoptosis in vitro and in vivo. **a** and **b** EdU assay and **c** CCK-8 assay determined cell proliferation of ZNF582-AS1-overexpressed OSRC2 and Caki-1 cells comparing with their control cells. **d** and **e** TUNEL assay and **f** and **g** flow cytometry determined cell apoptosis of ZNF582-AS1-overexpressed OSRC2 and Caki-1 cells comparing with their control cells. **h** Tumors collected from mice are shown. **i** and **j** Tumor volume curves and tumor weights of the ZNF582-AS1-overexpressed and control groups were measured and compared. **(k and l)** The cell proliferation and apoptosis of tumors were examined

RETRACTED

### ZNF582-AS1 overexpression inhibited cell migratory and invasive ability in vitro and in vivo

Compared with the control cells, the migratory and invasive abilities of ZNF582-AS1-overexpressed OSRC2 and Caki-1 cells were significantly decreased. Results showed that migratory distances of the ZNF582-AS1-overexpressed cells were significantly inhibited (Fig. 4a, b). The results of transwell migratory and invasive assays also indicated that migratory and invasive cells were significantly decreased in OSRC2 and Caki-1 cells that overexpressed ZNF582-AS1, compared with the control cells (Fig. 4c, d, e, f). To verify the inhibitory effect of ZNF582-AS1 on cell migration and invasion, in vivo mice model of metastasis was established. Metastasis experiments results confirmed that ZNF582-AS1 overexpression inhibited cancer cells metastasis to lung (Fig. 4g, h). There was no significant difference between the mouse weight of ZNF582-AS1-overexpressed and control groups (Fig. 4i). Haematoxylin-eosin staining was performed on the lung tissue to observe the metastases in the two groups. We found that ZNF582-AS1 overexpression significantly reduced the number and size of pulmonary metastases (Fig. 4j, k). EMT (Epithelial-mesenchymal transition) is one of the main pathways that regulates cancer cells invasion and migration [25]. Our results also showed that ZNF582-AS1 overexpression increased E-cadherin expression and decreased N-cadherin expression in pulmonary metastases (Fig. 4 l, m).

**Fig. 4:** ZNF582-AS1 overexpression inhibited cell migratory and invasive ability in vitro and in vivo. **a** and **b** Wound healing assay determined the migratory distances of ZNF582-AS1-overexpressed OSRC2 and Caki-1 cells and their control cells. **c** and **d** Transwell migration and **e** and **f** invasion assays determined the migratory and invasive abilities of ZNF582-AS1-overexpressed OSRC2 and Caki-1 cells and their control cells. **g** and **h** The luciferase signals in the ZNF582-AS1-overexpressed group were remarkably lower than those in the control group. **i** There was no significant difference between the mice weight of ZNF582-AS1-overexpressed and control group. **j** and **k** The number and size of pulmonary metastases in the ZNF582-AS1-overexpressed group were significantly reduced compared with those in the control group. **l** and **m** ZNF582-AS1 overexpression increased E-cadherin expression and decreased N-cadherin expression in pulmonary metastases

RETRACTED

### ZNF582-AS1 overexpression decreased rRNA adenine N(6)-methyltransferase A8K0B9 protein expression

To investigate the molecular mechanism of ZNF582-AS1 and identify its downstream targets in ccRCC, iTRAQ was performed to examine the expression changes at protein levels between the stable ZNF582-AS1-overexpressed OSRC2 cells and the control cells. The overexpression efficiency of ZNF582-AS1 in OSRC2 cell was shown in Fig. 5a. According to the ANOVA analysis results, 69 proteins were downregulated and 75 proteins were upregulated in ZNF582-AS1-overexpressed OSRC2 cells compared with control OSRC2 cells (Fig. 5b). These differently expressed proteins could remarkably separate ZNF582-AS1-overexpressed OSRC2 cells from the control cells (Fig. 5c). Biological Process GO term enrichment analysis of the complete 144 statistically significant proteins revealed “rRNA (adenine-N6,N6-)-dimethyltransferase activity”, “metalloendopeptidase inhibitor activity”, “rRNA (adenine) methyltransferase activity”, “RNA methyltransferase activity”, “catalytic activity, acting on a Rrna” and “rRNA methyltransferase activity” as the most significantly 6 enriched terms (Fig. 5d, Table 3). Interestingly, rRNA adenine N(6)-methyltransferase A8K0B9 and B4DRY2 proteins were involved in 5 of the 6 GO terms, suggesting A8K0B9 and B4DRY2 might be potential downstream targets of ZNF582-AS1.

**Fig. 5:** ZNF582-AS1 overexpression decreased rRNA adenine N(6)-methyltransferase A8K0B9 expression. **a** The overexpression efficiency of ZNF582-AS1 in OSRC2 cells. **b** iTRAQ results showed that 69 proteins were downregulated and 75 proteins were upregulated in ZNF582-AS1-overexpressed OSRC2 cells compared with control OSRC2 cells. **c** The expression of these 144 differently expressed proteins in ZNF582-AS1-overexpressed OSRC2 cells and control cells. **d** Biological Process GO term enrichment analysis of the complete 144 statistically significant proteins. **e** and **f** Validation of the presence of A8K0B9 protein. **g** A8K0B9 expression was decreased in ZNF582-AS1-overexpressed OSRC2 cells compared with control cells. **h** Changes of A8K0B9 protein level in OSRC2 cells after transient transfection of different doses of ZNF582-AS1 overexpression plasmid. **i** Estimation of the binding propensity of A8K0B9-ZNF582-AS1 pair. **j** RNA pull-down assay indicated that A8K0B9 protein bound specifically to ZNF582-AS1

**Table 3:** Biological Process GO term enrichment analysis of the complete 144 statistically significant proteins

Term	Description	***P***-value	Protein involve
GO:0000179	rRNA (adenine-N6,N6-)-	0.002118779	A8K0B9,B4DRY2
dimethyltransferase activity			
GO:0008191	metalloendopeptidase inhibitor activity	0.002118779	Q9BS40,Q5H9B4
GO:0016433	rRNA (adenine) methyltransferase activity	0.002118779	A8K0B9,B4DRY2
GO:0008173	RNA methyltransferase activity	0.006599965	A8K0B9,B4DRY2,Q8N1G2
GO:0140102	catalytic activity, acting on a rRNA	0.01195334	A8K0B9,B4DRY2
GO:0008649	rRNA methyltransferase activity	0.01195334	A8K0B9,B4DRY2
GO:0008081	phosphoric diester hydrolase activity	0.03817819	H0YJ44,Q15147
GO:0051723	protein methylesterase activity	0.04618345	Q9Y570
GO:0004706	JUN kinase kinase kinase activity	0.04618345	Q13546
GO:0017154	semaphorin receptor activity	0.04618345	E2PU09
GO:0051731	polynucleotide 5′-hydroxyl-kinase	0.04618345	Q5SY16
activity			
GO:0004181	metallocarboxypeptidase activity	0.04618345	O75976
GO:0004174	electron-transferring-flavoprotein	0.04618345	Q9BRQ8
dehydrogenase activity			
GO:0004483	mRNA (nucleoside-2′-O-)-	0.04618345	Q8N1G2
methyltransferase activity			
GO:0051722	protein C-terminal	0.04618345	Q9Y570
methylesterase activity			
GO:0033981	D-dopachrome decarboxylase activity	0.04618345	P30046
GO:0061501	cyclic-GMP-AMP synthase activity	0.04618345	Q8N884
GO:0005225	volume-sensitive anion	0.04618345	Q8TDW0
channel activity			
GO:0016649	oxidoreductase activity,	0.04618345	Q9BRQ8
acting on the CH-NH group of donors,			
quinone or similar compound as acceptor			
GO:0050023	L-fuconate dehydratase activity	0.04618345	J3QL81

However, the UniProt database (https://www.uniprot.org/uniprot/) showed that A8K0B9 (predicted mass: 39.538 KD) and B4DRY2 (predicted mass: 27.265 KD) have only been validated at the transcription level. To prove the existence of the two proteins, recombinant pLV-hef1a-mNeongreen-P2A-Puro-WPRE-CMV-B4DRY2-3Xflag and pLV-hef1a-mNeongreen-P2A-Puro-WPRE-CMV-A8K0B9-3Xflag plasmid vectors were constructed, and the western blot results verified the presence of A8K0B9 protein (Fig. 5e). Since A8K0B9 has a 90% identity with TFB1M protein which has been validated at protein level (Additional file 5: Figure S4), TFB1M antibody (Sigma) targeted the consensus protein sequences of A8K0B9 and TFB1M was used to detect the sum protein expression of A8K0B9 and TFB1M in ZNF582-AS1-overexpressed and control OSRC2 cells, and another TFB1M antibody (Abcam) only target TFB1M protein was used to examine the expression of TFB1M. Western Blot results showed that TFB1M was expressed equally in A8K0B9-overexpressed OSRC2 cells and control cells, while the sum protein expression of A8K0B9 and TFB1M was increased in A8K0B9-overexpressed OSRC2 cells compared with control cells (Fig. 5f). Then, we examined the expression of A8K0B9 protein in ZNF582-AS1-overexpressed and control OSRC2 cells, and results demonstrated that TFB1M was expressed equally in ZNF582-AS1-overexpressed OSRC2 cells and control cells, while the sum protein expression of A8K0B9 and TFB1M was decreased in ZNF582-AS1-overexpressed OSRC2 cells compared with control cells, suggesting the decreased A8K0B9 protein expression in ZNF582-AS1-overexpressed OSRC2 cells (Fig. 5g). Moreover, after transiently transfecting different doses of ZNF582-AS1 overexpression plasmid into OSRC2 cells, we also found that the expression of A8K0B9 protein decreased with the increase of ZNF582-AS1 expression (Fig. 5h).

RETRACTED

To investigate whether A8K0B9 protein could bind to ZNF582-AS1. catRAPID, an algorithm, was used to estimate the binding propensity of A8K0B9-ZNF582-AS1 pair. Evaluation results indicated that A8K0B9 and ZNF582-AS1 have a certain binding propensity (Fig. 5i, Additional file 6: Figure S5). Moreover, in vitro RNA pull-down assay with biotinylated ZNF582-AS1 and antisense control RNA was performed to confirm the binding between ZNF582-AS1 RNA and A8K0B9 protein. Western blot analysis of ZNF582-AS1-enriched proteins after RNA pull-down indicated that A8K0B9 protein bound specifically to ZNF582-AS1 RNA (Fig. 5j).

### ZNF582-AS1 regulated the N(6)-methyladenosine modification of MT-RNR1 by modulating A8K0B9

Since ZNF582-AS1 could bind with A8K0B9 to induce its downregulation, we wondered whether ZNF582-AS1 could regulate the N(6)-methyladenosine modification of rRNA. We performed the rRNA MeRIP-seq to identify the differentially methylated rRNA sites between ZNF582-AS1-overexpressed and control OSRC2 cells, and the unmodified_Control_RNA and m6A_Control_RNA were used as negative and positive controls, respectively (Fig. 6a). The rRNA MeRIP-seq results showed that the methylation levels of 3 and 4 peaks of MT-RNR2 were upregulated and downregulated in ZNF582-AS1-overexpressed OSRC2 cells compared with control OSRC2 cells, respectively. The methylation levels of a peak of RNA28SN5 and a peak of MT-RNR1 were upregulated and downregulated in ZNF582-AS1-overexpressed OSRC2 cells, respectively (Fig. 6b). Then, we examined MT-RNR1, MT-RNR2 and RNA28SN5 expression in ZNF582-AS1-overexpressed and control OSRC2 cells by qRT-PCR. Our results indicated that only the expression of MT-RNR1 was significantly changed in ZNF582-AS1-overexpressed OSRC2 cells compared with control OSRC2 cells (Fig. 6c). Consistent with our results, MT-RNR1 expression was negatively associated with ZNF582-AS1 expression, and lower MT-RNR1 expression was related to longer OS based on TCGA-KIRC data (Fig. 6d, e). We also tested the expression of MT-RNR1 in ccRCC cell lines, and the results showed that compared with HK2 cells, MT-RNR1 expression was significantly increased in OSRC2 and Caki-1 cells with higher DNA methylation level of ZNF582-AS1 promoter (Fig. 6f).

RETRACTED

**Fig. 6:** ZNF582-AS1 regulated the N(6)-methyladenosine modification of MT-RNR1 by modulating A8K0B9. **a** Negative and positive controls of rRNA MeRIP-seq. **b** The analysis results of rRNA MeRIP-seq. **c** The expression of MT-RNR1, MT-RNR2 and RNA28SN5 in ZNF582-AS1-overexpressed and control OSRC2 cells. **d** and **e** MT-RNR1 expression was negatively associated with ZNF582-AS1 expression (*n* = 530), and lower MT-RNR1 expression was related to longer OS (n = 530) based on TCGA-KIRC data. According to the median cutoff of MT-RNR1 expression, patients were divided into two groups for survival analysis. **f** The expression of MT-RNR1 in ccRCC cell lines. **g** Analysis of m6A motif DRACH (D = A, G or U; R = A or G; H = A, U or C) in MT-RNR1 sequence. **h** MeRIP-qPCR determined the methylation level of MT-RNR1 in ZNF582-AS1-overexpressed OSRC2 cells and control cells. **i** RIP-RT-qPCR showed that A8K0B9 protein had a certain binding ability with MT-RNR1 in OSRC2 cells

To further determine the regulation mechanism of ZNF582-AS1 on MT-RNR1, analysis of m6A motif DRACH (D = A, G or U; R = A or G; H = A, U or C) indicated that there were 2 motifs in MT-RNR1 (Fig. 6g), and the MeRIP-qPCR results also showed that the methylation level of MT-RNR1 was significantly decreased in ZNF582-AS1-overexpressed OSRC2 cells (Fig. 6h). Furthermore, the results of RIP-qRT-PCR showed that A8K0B9 protein had a certain binding ability with MT-RNR1 in OSRC2 cells (Fig. 6i). Taken together, our results confirmed that ZNF582-AS1 could regulate the N(6)-methyladenosine modification of MT-RNR1 by modulating A8K0B9 protein.

### ZNF582-AS1 overexpression decreased MT-CO2 protein expression by regulating MT-RNR1

Mitochondrial gene expression requires a series of interrelated processes, including mitochondrial DNA (mtDNA) replication and repair, mitochondrial RNA transcription, maturation, and mitochondrial glycosome assembly [26]. Based on the above results, we have determined that MT-RNR1 expression was dysregulated in ZNF582-AS1-overexpressed ccRCC cells. So, does the dysregulation expression of MT-RNR1 cause related changes in mitochondrial protein expression? The human mitochondrial genome encodes 13 subunits of respiratory chain complexes: seven subunits (ND 1–6 and 4 L) of complex I, cytochrome b (Cyt b) of complex III, the COX I–III subunits of cytochrome oxidase or complex IV, and the ATPase 6 and 8 subunits of F(o)F(1)-ATP synthase. Based on the TCGA-KIRC data, the expression of all these 13 genes (MT-ND1, MT-ND2, MT-ND3, MT-ND4, MT-ND5, MT-ND6, MT-ND4L, MT-CYB, MT-CO1, MT-CO2, MT-CO3, MT-ATP6 and MT-ATP8) was positively correlated with MT-RNR1 expression (Additional file 7: Figure S6). Among them, MT-CO2 (mitochondrially encoded cytochrome c oxidase II) has the highest correlation with MT-RNR1 (Fig. 7a). Besides, lower MT-CO2 expression was associated with longer OS based on TCGA-KIRC data (Fig. 7b), and the iTRAQ results indicated that MT-CO2 (A0A0P0C1B5) protein expression was decreased in ZNF582-AS1-overexpressed OSRC2 cells compared with control OSRC2 cells (Fig. 7c). Moreover, our results found that MT-CO2 protein expression was decreased in ZNF582-AS1-overexpressed OSRC2 cells compared with control OSRC2 cells (Fig. 7d, e). As the center of cellular bioenergetics, with numerous metabolic pathways and signaling cascades, the health of mitochondria is critical to ensuring cell survival. It was reported that mitochondrial proteins play important roles in various biological activities, such as energy homeostasis and apoptosis [27]. Due to the unique physiological characteristics of mitochondria, they are constantly being destroyed by destructive oxidative stress, and oxidative stress can cause changes in mitochondrial dynamics, which in turn leads to increased reactive oxygen species (ROS) production, leading to abnormal mitochondrial function [27, 28]. In this study, our results found that the expression of Bcl-2 and N-cadherin protein was decreased, while Cleaved Caspase 3 and E-cadherin protein expression and ROS levels were increased in ZNF582-AS1-overexpressed OSRC2 cells compared with control OSRC2 cells (Fig. 7d, e, f, g).

RETRACTED

**Fig. 7:** ZNF582-AS1 overexpression decreased MT-CO2 expression by regulating MT-RNR1. **a** and **b** MT-CO2 expression was significantly positively correlated with MT-RNR1 expression (n = 530), and lower MT-CO2 expression was associated with longer OS (n = 530) based on TCGA-KIRC data. According to the median cutoff of MT-CO2 expression, patients were divided into two groups for survival analysis. **c** Based on the iTRAQ results, the expression level of MT-CO2 (A0A0P0C1B5) protein was decreased in ZNF582-AS1-overexpressed OSRC2 cells compared with control OSRC2 cells. **d** and **e** MT-CO2, Bcl-2 and N-cadherin protein expression was decreased and Cleaved Caspase 3 and E-cadherin protein expression was increased in ZNF582-AS1-overexpressed OSRC2 cells compared with control cells. **f** and **g** The ROS level in ZNF582-AS1-overexpressed OSRC2 cells was increased. **h** The overexpression efficiency of MT-RNR1 in ZNF582-AS1-overexpressed OSRC2 cells. **i** and **j** MT-CO2, Bcl-2 and N-cadherin protein expression was increased and Cleaved Caspase 3 and E-cadherin protein expression was decreased in MT-RNR1-overexpressed-ZNF582-AS1-overexpressed OSRC2 cells compared with control cells. **k** and **l** The ROS level in MT-RNR1-overexpressed-ZNF582-AS1-overexpressed OSRC2 cells was decreased

To further determine whether ZNF582-AS1 overexpression reduced MT-CO2 expression by regulating MT-RNR1, recombinant pLV-hef1a-mNeongreen-P2A-Puro-WPRE-CMV-MT-RNR1 plasmid vector was constructed (Fig. 7h). Our results demonstrated that the expression of MT-CO2, Bcl-2 and N-cadherin protein was increased, while Cleaved Caspase 3 and E-cadherin protein expression and ROS levels were decreased in MT-RNR1-overexpressed-ZNF582-AS1-overexpressed OSRC2 cells compared with ZNF582-AS1-overexpressed OSRC2 cells (Fig. 7i, j, k, l). Taken together, the above findings identified that ZNF582-AS1 overexpression decreased MT-CO2 protein expression by regulating MT-RNR1.

RETRACTED

### MT-RNR1 overexpression reversed the inhibition of cell proliferative, migratory and invasive ability and the increase of cell apoptotic rate caused by ZNF582-AS1 overexpression in vitro and in vivo

Considering that ZNF582-AS1 overexpression decreases MT-CO2 expression by regulating MT-RNR1, the question is whether MT-RNR1 overexpression can reverses inhibited cell proliferative, migratory and invasive ability and increased cell apoptosis caused by ZNF582-AS1 overexpression. Our results showed that MT-RNR1 overexpression promoted cell proliferation (Fig. 8a, b, c) and inhibited cell apoptosis (Fig. 8d, e, f, g) in ZNF582-AS1-overexpressed OSRC2 and Caki-1 cells. Consistent with the increased proliferative ability and low apoptotic rate observed in the MT-RNR1-overexpressed-ZNF582-AS1-overexpressed OSRC2 and Caki-1 cells, the xenograft experiment in mice also found that MT-RNR1-overexpressed-ZNF582-AS1-overexpressed tumors grew faster than those in the control group (Fig. 8h, i, j). Moreover, the results of immunohistochemistry confirmed that overexpression of MT-RNR1 promoted cell proliferation and inhibited cell apoptosis in ZNF582-AS1-overexpressed tumors (Fig. 8k, l).

**Fig. 8:** MT-RNR1 overexpression reversed inhibited cell proliferation and increased cell apoptosis caused by ZNF582-AS1 overexpression. **a** and **b** EdU assay and **c** CCK-8 assay determined cell proliferation of MT-RNR1-overexpressed-ZNF582-AS1-overexpressed OSRC2 and Caki-1 cells comparing with their control cells. **d** and **e** TUNEL assay and **f** and **g** flow cytometry determined cell apoptosis of MT-RNR1-overexpressed-ZNF582-AS1-overexpressed OSRC2 and Caki-1 cells comparing with their control cells. **h** Tumors collected from mice are shown. **i** and **j** Tumor volume curves and tumor weights of the MT-RNR1-overexpressed-ZNF582-AS1-overexpressed and control groups were measured and compared. **k** and **l** The cell proliferation and apoptosis of tumor were examined

In addition, the migratory distances of the MT-RNR1-overexpressed-ZNF582-AS1-overexpressed group were significantly increased (Fig. 9a, b). Meanwhile, migratory and invasive cells were remarkably increased in ZNF582-AS1-overexpressed OSRC2 and Caki-1 cells that overexpressed MT-RNR1, compared with the control cells (Fig. 9c, d, e, f). Furthermore, mice metastasis experiments results indicated that MT-RNR1 overexpression increased the incidence of pulmonary metastasis (Fig. 9g, h). There was no significant difference between the mice weight of the two treatment group (Fig. 9i). Haematoxylin-eosin staining results determined that MT-RNR1 overexpression remarkably increased the number and size of pulmonary metastases (Fig. 9j, k). Besides, MT-RNR1 overexpression decreased E-cadherin expression and increased N-cadherin expression in pulmonary metastases (Fig. 9l, m). Taken together, our results demonstrated that MT-RNR1 overexpression could reverse the phenotype inhibition of ccRCC induced by increased ZNF582-AS1 expression. As shown in Fig. 10, ZNF582-AS1 overexpression suppresses the N(6)-methyladenosine modification of MT-RNR1 by reducing A8K0B9 protein level, resulting in the decrease of MT-RNR1 and MT-CO2 expression and subsequently phenotype inhibition of ccRCC cells, thus playing the role of tumor suppressor gene in ccRCC pathogenesis.

RETRACTED

**Fig. 9:** MT-RNR1 overexpression reversed inhibited cell migratory and invasive ability caused by ZNF582-AS1 overexpression. **a** and **b** Wound healing assay determined the migratory distances of MT-RNR1-overexpressed-ZNF582-AS1-overexpressed OSRC2 and Caki-1 cells and their control cells. **c** and **d** Transwell migration and **e** and **f** invasion assays determined the migratory and invasive abilities of MT-RNR1-overexpressed-ZNF582-AS1-overexpressed OSRC2 and Caki-1 cells and their control cells. **g** and **h** The luciferase signals in the MT-RNR1-overexpressed-ZNF582-AS1-overexpressed group were remarkably higher than those in the ZNF582-AS1-overexpressed group. **i** There was no significant difference between the mouse weight of the two treatment group. **j** and **k** The number and size of pulmonary metastases in the MT-RNR1-overexpressed-ZNF582-AS1-overexpressed group were significantly increased compared with those in the ZNF582-AS1-overexpressed group. **l** and **m** MT-RNR1 overexpression decreased E-cadherin expression and increased N-cadherin expression in pulmonary metastases

**Fig. 10:** Schematic diagram of the tumor suppressor effect of ZNF582-AS1 in ccRCC

RETRACTED

## Discussion

LncRNAs with a length of more than 200 nucleotides have been shown to function as oncogenes or tumor suppressor genes in the process of tumorigenesis [29]. In addition to their functional effects on tumor progression, lncRNAs also display various regulatory effects through different mechanisms, including regulation of mRNA processing and translation, epigenetic transcriptional modulation, remodeling of and interactions with chromatin, genome defense or RNA turnover [30]. Besides, lncRNAs expression has been quantitatively studied in several tumor cell types and tissues by high-throughput RNA sequencing (RNA-seq) and have commonly been found to be more tumor cell type specific than the expression of protein-coding genes [31]. Moreover, many studies have also suggested that lncRNAs abnormal expression is responsible for drug resistance, which is a major obstacle for tumor treatment [18, 32]. Therefore, lncRNAs have been considered not only as potential molecular biomarkers, but also as significantly therapeutic targets for tumor treatment.

Recent advancements in the rapidly evolving field of cancer epigenetics have shown extensive reprogramming of every component of the epigenetic machinery in RCC, including DNA methylation, histone modification and nucleosomal localization [33]. DNA methylation was one of the first modes of epigenetic regulation to be discovered, and alterations in DNA methylation have also been examined in ccRCC [34]. Numerous tumor suppressor genes have been reported to be partially or completely silenced due to hypermethylation of their promoters in single-locus studies, and the use of hypomethylating agents has been shown to restore the expression of many of these genes in vitro [35]. ZNF582-AS1 is a newly identified lncRNA that has been mapped to the human chromosome 19q13.43, and it is differentially expressed in ccRCC and exhibit diagnostic and prognostic values in ccRCC [21]. Besides, study indicated that ZNF582-AS1 is epigenetically silenced by aberrant DNA methylation in colorectal cancer [22]. However, most of these results are obtained by analyzing the TCGA data, and no experimental study has explored the specific role and mechanism of ZNF582-AS1 in ccRCC so far.

During our study, we found that ZNF582-AS1 expression was significantly downregulated in ccRCC tissues and cells, and decreased ZNF582-AS1 expression was significantly associated with advanced tumor stage, higher pathological stage, distant metastasis, and poor prognosis. Besides, the RNA FISH results showed that ZNF582-AS1 was distributed mostly in the cytoplasm of ccRCC cells. Bioinformatic data mining found DNA hypermethylation in the promoter ZNF582-AS1 DNA, and the expression of ZNF582-AS1 was negatively correlated with the methylation status of its CpG sites. Meanwhile, higher methylation levels of these CpG sites were significantly associated with ccRCC progression and poor prognosis. In addition, our MSP and Sequenom MassARRAY results confirmed the hypermethylation status of ZNF582-AS1 in ccRCC tissues and cells, and treatment with 5-Aza and TSA induced demethylation of the ZNF582-AS1 promoter and increased ZNF582-AS1 expression. Furthermore, in vitro and in vivo assays both found that ZNF582-AS1 overexpression significantly inhibited cell proliferation and induced cell apoptosis. Cell migratory and invasive abilities were also suppressed by ZNF582-AS1 overexpression. Interestingly, previous studies indicated that ZNF582-AS1 does not affect cell viability or proliferation, the cell cycle or apoptosis in CRC cell lines [22]. Therefore, ZNF582-AS1 may act in different ways in different tumors, and its role in other tumors needs further study.

RETRACTED

To explore the molecular mechanisms of the tumor suppressive function of ZNF582-AS1 in ccRCC, iTRAQ analysis and RNA pull down assays were performed to identify the downstream targets of ZNF582-AS1. Results showed that ZNF582-AS1 was able to bind with A8K0B9 protein (rRNA adenine N(6)-methyltransferase) and caused its degradation, which indicates that ZNF582-AS1 may modulate the N(6)-methyladenosine modification of rRNA in ccRCC. N(6)-methyladenosine is one of the most common RNA modifications in eukaryotes, mainly in mRNA [36]. Recent studies have discovered a number of lncRNAs modified by N(6)-methyladenosine in multiple cancers, and they can regulate gene expression and function through a series of complex mechanisms [37–42]. In turn, lncRNAs can target or modulate N(6)-methyladenosine regulators to influence the development of cancer [43]. However, the role of lncRNAs in the N(6)-methyladenosine modification of rRNA remains unknown. In this study, our results showed that the N(6)-methyladenosine modification level of MT-RNR1 was downregulated in ZNF582-AS1-overexpressed OSRC2 cells compare with control OSRC2 cells, and the expression of MT-RNR1 in ZNF582-AS1-overexpressed OSRC2 cells was decreased. Moreover, A8K0B9 protein had a certain binding ability with MT-RNR1 in OSRC2 cells. It was reported that binding of YTHDF2 (the human YTH domain family 2), a N(6)-methyladenosine “reader” protein, results in the localization of bound mRNA from the translatable pool to mRNA decay sites, such as processing bodies, thereby promoting mRNA degradation [44]. However, in the present study, we found that reduced N(6)-methyladenosine modification level of MT-RNR1 caused a reduction in MT-RNR1 expression. In order to clarify this inconsistency, more studies are needed in the near future to identify the specific effect of N(6)-methyladenosine modification on rRNA expression.

RETRACTED

Mitochondria are organelles that perform major roles in cellular operation. Therefore, alterations in mitochondrial genome may lead to mitochondrial dysfunction and cellular deregulation, influencing carcinogenesis [45]. A recent study indicated that ZCCHC4 is a new human N(6)-methyladenosine methyltransferase, and knockout of ZCCHC4 eliminates the N(6)-methyladenosine modification on 28S rRNA, thereby reducing overall translation activity, which contributes to inhibiting liver cancer cells proliferation and reducing liver tumor size [46]. In the current study, our results demonstrated that MT-CO2 expression was positively correlated with MT-RNR1 expression, and ZNF582-AS1 overexpression decreased the expression of MT-CO2 protein. Previous studies have shown that elevated mitochondrial protein Lon promotes EMT via reactive oxygen species (ROS)-dependent signaling [47]. Studies also indicated that MRC proteins including MT-CO2 are induced early before ROS and apoptosis of multiple cell types induced by multiple stimuli [48, 49]. Consistent with the above findings, our results showed that the expression of Bcl-2 and N-cadherin protein was decreased, while Cleaved Caspase 3 and E-cadherin protein expression and ROS levels were increased in ZNF582-AS1-overexpressed OSRC2 cells. Moreover, our results demonstrated that MT-RNR1 overexpression rescued the decreased expression of MT-CO2, Bcl-2 and N-cadherin and the increased expression of Cleaved Caspase 3 and E-cadherin and ROS levels caused by ZNF582-AS1 overexpression. Furthermore, MT-RNR1 overexpression reversed decreased cell proliferative, migratory and invasive ability and increased cell apoptotic rate caused by ZNF582-AS1 overexpression in vitro and in vivo.

## Conclusions

Our results revealed that lncRNA ZNF582-AS1 expression is silenced by abnormal DNA hypermethylation in promoter. ZNF582-AS1 overexpression inhibits cell proliferative, migratory and invasive ability and promotes cell apoptosis in ccRCC through suppressing the N(6)-methyladenosine modification of MT-RNR1, resulting in the decrease of MT-RNR1 expression, followed by the decrease of MT-CO2 protein. The results of this study provide a new basis for studying the mechanism of the progression and metastasis of ccRCC. Cumulatively, our results demonstrates for the first time that ZNF582-AS1 functions as a tumor suppressor gene in ccRCC, and ZNF582-AS1 may serve as a potential prognostic biomarker and therapeutic target of ccRCC.

RETRACTED

## Supplementary Information

**Additional file 1: Table S1.** The detailed primers information of qRT-PCR, MSP, Sequenom MassARRAY quantitative methylation analysis and MeRIP-qRT-PCR.

**Additional file 2: Figure S1.** ZNF582-AS1 promoter high DNA methylation level is associated with low ZNF582-AS1 expression in ccRCC. (a) Heatmap and statistical comparison (b) of the difference in the methylation levels of 13 CpG sites in ccRCC (*n* = 325) and adjacent normal renal tissues (*n* = 160). (c) The negative correlation between ZNF582-AS1 methylation status and ZNF582-AS1 expression (*n* = 317).

**Additional file 3: Figure S2.** The correlation between ZNF582 expression and the methylation levels of 13 CpG sites (n = 317).

**Additional file 4: Figure S3.** The prognostic roles of the methylation levels of ZNF582-AS1 CpG sites in ccRCC patients. (a) The association between the methylation levels of ZNF582-AS1 CpG sites and OS (n = 317). (b) The association between the methylation levels of ZNF582-AS1 CpG sites and DFS (*n* = 280). According to the median cutoff of the methylation levels of CpG sites, patients were divided into two groups for survival analysis.

**Additional file 5: Figure S4.** Comparison of A8K0B9 and TFB1M protein sequences.

**Additional file 6: Figure S5.** Estimation of the binding propensity of A8K0B9-ZNF582-AS1 pair.

**Additional file 7: Figure S6.** The correlation between MT-RNR1 expression and the mRNA expression of 12 mitochondrial proteins (n = 317).

## Data Availability

The datasets used and/or analyzed during the current study are available from the corresponding author on reasonable request.

## Abbreviations

ccRCC: Clear cell renal cell carcinoma
OS: Overall Survival
DFS: Disease Free Survival
qRT-PCR: Quantitative real-time PCR
TCGA-KIRC: The Cancer Genome Atlas-Kidney Renal Clear Cell Carcinoma
MSP: Methylation-specific PCR
EdU: Ethynyl-2-deoxyuridine
iTRAQ: Isotope Tagging for Relative and Absolute protein Quantitation
RIP: RNA immunoprecipitation
ROS: Reactive oxygen species
MRC: Mitochondrial respiratory chain
EMT: Epithelial-mesenchymal transition

## References

[1] Bray F, Ferlay J, Soerjomataram I, Siegel RL, Torre LA, Jemal A (2018). Global cancer statistics 2018: GLOBOCAN estimates of incidence and mortality worldwide for 36 cancers in 185 countries. CA Cancer J Clin.

[2] Frank I, Blute ML, Leibovich BC, Cheville JC, Lohse CM, Zincke H (2005). Independent validation of the 2002 American joint committee on cancer primary tumor classification for renal cell carcinoma using a large, single institution cohort. J Urol.

RETRACTED

[3] Choueiri TK, Motzer RJ (2017). Systemic therapy for metastatic renal-cell carcinoma. N Engl J Med.

[4] Hsieh JJ, Purdue MP, Signoretti S, Swanton C, Albiges L, Schmidinger M (2017). Renal cell carcinoma. Nat Rev Dis Prim.

[5] Barata PC, Rini BI (2017). Treatment of renal cell carcinoma: current status and future directions. CA Cancer J Clin.

[6] Reustle A, Di Marco M, Meyerhoff C, Nelde A, Walz JS, Winter S (2020). Integrative -omics and HLA-ligandomics analysis to identify novel drug targets for ccRCC immunotherapy. Genome Med.

[7] Deveson IW, Hardwick SA, Mercer TR, Mattick JS (2017). The dimensions, dynamics, and relevance of the mammalian noncoding Transcriptome. Trends Genetics.

[8] Esposito R, Bosch N, Lanzos A, Polidori T, Pulido-Quetglas C, Johnson R (2019). Hacking the Cancer genome: profiling therapeutically actionable long non-coding RNAs using CRISPR-Cas9 screening. Cancer Cell.

[9] Slack FJ, Chinnaiyan AM (2019). The role of non-coding RNAs in oncology. Cell..

[10] Peng WX, Koirala P, Mo YY (2017). LncRNA-mediated regulation of cell signaling in cancer. Oncogene..

[11] Wang G, Zhang ZJ, Jian WG, Liu PH, Xue W, Wang TD (2019). Novel long noncoding RNA OTUD6B-AS1 indicates poor prognosis and inhibits clear cell renal cell carcinoma proliferation via the Wnt/beta-catenin signaling pathway. Mol Cancer.

[12] Hamilton MJ, Young M, Jang K, Sauer S, Neang VE, King AT (2020). HOTAIRM1 lncRNA is downregulated in clear cell renal cell carcinoma and inhibits the hypoxia pathway. Cancer Lett.

[13] Zhai W, Zhu R, Ma J, Gong D, Zhang H, Zhang J (2019). A positive feed-forward loop between LncRNA-URRCC and EGFL7/P-AKT/FOXO3 signaling promotes proliferation and metastasis of clear cell renal cell carcinoma. Mol Cancer.

[14] Li JK, Chen C, Liu JY, Shi JZ, Liu SP, Liu B (2017). Long noncoding RNA MRCCAT1 promotes metastasis of clear cell renal cell carcinoma via inhibiting NPR3 and activating p38-MAPK signaling. Mol Cancer.

[15] Shen H, Laird PW (2013). Interplay between the cancer genome and epigenome. Cell..

[16] Amin V, Harris RA, Onuchic V, Jackson AR, Charnecki T, Paithankar S (2015). Epigenomic footprints across 111 reference epigenomes reveal tissue-specific epigenetic regulation of lincRNAs. Nat Commun.

[17] Wang Z, Yang B, Zhang M, Guo W, Wu Z, Wang Y (2018). lncRNA Epigenetic Landscape Analysis Identifies EPIC1 as an Oncogenic lncRNA that Interacts with MYC and Promotes Cell-Cycle Progression in Cancer. Cancer Cell.

[18] Lu C, Wei Y, Wang X, Zhang Z, Yin J, Li W (2020). DNA-methylation-mediated activating of lncRNA SNHG12 promotes temozolomide resistance in glioblastoma. Mol Cancer.

RETRACTED

[19] Wang B, Zhao L, Chi W, Cao H, Cui W, Meng W (2019). Aberrant methylation-mediated downregulation of lncRNA SSTR5-AS1 promotes progression and metastasis of laryngeal squamous cell carcinoma. Epigenetics Chromatin.

[20] Xu H, Sun Y, Ma Z, Xu X, Qin L, Luo B (2018). LOC134466 methylation promotes oncogenesis of endometrial carcinoma through LOC134466/hsa-miR-196a-5p/TAC1 axis. Aging..

[21] Cheng G, Liu D, Liang H, Yang H, Chen K, Zhang X (2019). A cluster of long non-coding RNAs exhibit diagnostic and prognostic values in renal cell carcinoma. Aging..

[22] Kumegawa K, Maruyama R, Yamamoto E, Ashida M, Kitajima H, Tsuyada A (2016). A genomic screen for long noncoding RNA genes epigenetically silenced by aberrant DNA methylation in colorectal cancer. Sci Rep.

[23] Carlevaro-Fita J, Johnson R (2019). Global positioning system: understanding long noncoding RNAs through subcellular localization. Mol Cell.

[24] Sharma S, Kelly TK, Jones PA (2010). Epigenetics in cancer. Carcinogenesis..

[25] Wang G, Zhang ZJ, Jian WG, Liu PH, Xue W, Wang TD (2019). Novel long noncoding RNA OTUD6B-AS1 indicates poor prognosis and inhibits clear cell renal cell carcinoma proliferation via the Wnt/β-catenin signaling pathway. Mol Cancer.

[26] Chen H, Shi Z, Guo J, Chang KJ, Chen Q, Yao CH (2020). The human mitochondrial 12S rRNA m(4)C methyltransferase METTL15 is required for mitochondrial function. J Biol Chem.

[27] Singh RK, Saini SK, Prakasam G, Kalairasan P, Bamezai RNK (2019). Role of ectopically expressed mtDNA encoded cytochrome c oxidase subunit I (MT-COI) in tumorigenesis. Mitochondrion..

[28] Sulkshane P, Duek I, Ram J, Thakur A, Reis N, Ziv T (2020). Inhibition of proteasome reveals basal mitochondrial ubiquitination. J Proteome.

[29] Bach DH, Lee SK (2018). Long noncoding RNAs in cancer cells. Cancer Lett.

[30] Prensner JR, Chinnaiyan AM (2011). The emergence of lncRNAs in cancer biology. Cancer Discov.

[31] Fatica A, Bozzoni I (2014). Long non-coding RNAs: new players in cell differentiation and development. Nat Rev Genet.

[32] Yu AM, Ingelman-Sundberg M, Cherrington NJ, Aleksunes LM, Zanger UM, Xie W (2017). Regulation of drug metabolism and toxicity by multiple factors of genetics, epigenetics, lncRNAs, gut microbiota, and diseases: a meeting report of the 21(st) international symposium on Microsomes and drug oxidations (MDO). Acta Pharm Sin B.

[33] Joosten SC, Smits KM, Aarts MJ, Melotte V, Koch A, Tjan-Heijnen VC (2018). Epigenetics in renal cell cancer: mechanisms and clinical applications. Nat Rev Urol.

[34] Lasseigne BN, Brooks JD (2018). The role of DNA methylation in renal cell carcinoma. Mol Diagnosis Ther.

RETRACTED

[35] Shenoy N, Vallumsetla N, Zou Y, Galeas JN, Shrivastava M, Hu C (2015). Role of DNA methylation in renal cell carcinoma. J Hematol Oncol.

[36] Boccaletto P, Machnicka MA, Purta E, Piatkowski P, Baginski B, Wirecki TK (2018). MODOMICS: a database of RNA modification pathways. 2017 update. Nucleic Acids Res.

[37] Zhou KI, Parisien M, Dai Q, Liu N, Diatchenko L, Sachleben JR (2016). N(6)-Methyladenosine Modification in a Long Noncoding RNA Hairpin Predisposes Its Conformation to Protein Binding. J Mol Biol.

[38] Yang D, Qiao J, Wang G, Lan Y, Li G, Guo X (2018). N6-Methyladenosine modification of lincRNA 1281 is critically required for mESC differentiation potential. Nucleic Acids Res.

[39] Yang X, Zhang S, He C, Xue P, Zhang L, He Z (2020). METTL14 suppresses proliferation and metastasis of colorectal cancer by down-regulating oncogenic long non-coding RNA XIST. Mol Cancer.

[40] Zuo X, Chen Z, Gao W, Zhang Y, Wang J, Wang J (2020). M6A-mediated upregulation of LINC00958 increases lipogenesis and acts as a nanotherapeutic target in hepatocellular carcinoma. J Hematol Oncol.

[41] Zhang S, Zhao BS, Zhou A, Lin K, Zheng S, Lu Z (2017). m(6)A Demethylase ALKBH5 Maintains Tumorigenicity of Glioblastoma Stem-like Cells by Sustaining FOXM1 Expression and Cell Proliferation Program. Cancer cell.

[42] Hu X, Peng WX, Zhou H, Jiang J, Zhou X, Huang D (2020). IGF2BP2 regulates DANCR by serving as an N6-methyladenosine reader. Cell Death Differ.

[43] Yi YC, Chen XY, Zhang J, Zhu JS (2020). Novel insights into the interplay between m(6)a modification and noncoding RNAs in cancer. Mol Cancer.

[44] Wang X, Lu Z, Gomez A, Hon GC, Yue Y, Han D (2014). N6-methyladenosine-dependent regulation of messenger RNA stability. Nature..

[45] Cavalcante GC, Marinho ANR, Anaissi AK, Vinasco-Sandoval T, Ribeiro-Dos-Santos A, Vidal AF (2019). Whole mitochondrial genome sequencing highlights mitochondrial impact in gastric cancer. Sci Rep.

[46] Ma H, Wang X, Cai J, Dai Q, Natchiar SK, Lv R (2019). N(6-)Methyladenosine methyltransferase ZCCHC4 mediates ribosomal RNA methylation. Nat Chem Biol.

[47] Kuo CL, Chou HY, Chiu YC, Cheng AN, Fan CC, Chang YN (2020). Mitochondrial oxidative stress by Lon-PYCR1 maintains an immunosuppressive tumor microenvironment that promotes cancer progression and metastasis. Cancer Lett.

[48] Chandra D, Liu JW, Tang DG (2002). Early mitochondrial activation and cytochrome c up-regulation during apoptosis. J Biol Chem.

[49] Chwa M, Atilano SR, Hertzog D, Zheng H, Langberg J, Kim DW (2008). Hypersensitive response to oxidative stress in keratoconus corneal fibroblasts. Invest Ophthalmol Vis Sci.

